The article "Analysis of the Factors Related to Intracranial Infection after Brain Tumor Surgery" was retracted in 2023. Reasons: unreliable results or conclusions; lack of ethics approval or compliance; concerns about the data; concerns about the peer review.

# Analysis of the Factors Related to Intracranial Infection after Brain Tumor Surgery

**DOI:** 10.1155/2022/6988560

**Published:** 2022-09-05

**Authors:** Weiying Chen, Danli Sheng

**Affiliations:** ^1^Oncology Department Zhejiang Hospital, Hangzhou 310030, China; ^2^Neurosurgery Department Zhejiang Hospital, Hangzhou 310030, China

## Abstract

In order to explore the factors related to intracranial infection after brain tumor surgery, a retrospective analysis is conducted in this study. According to the patients with intracranial infection after brain tumor surgery in our hospital from January 2020 to October 2020, clinical data are divided into different groups and some indicators are put into the multiple regression model for multivariate analysis. The factors related to intracranial infection after brain tumor surgery are analyzed, and the clinical effect of a detailed management plan based on the abovementioned risk factors to prevent intracranial infection in patients after brain tumor surgery is observed. Multiple regression models demonstrate that complicated underlying diseases, operation time, and intraoperative blood loss are independent risk factors for postoperative intracranial infection.

## 1. Introduction

As the general name of various tumors growing in the skull cavity, brain tumors can occur in the meninges, nerves, blood vessels, and various brain attachments. Some tumors may also be invaded and formed due to tumor metastasis in other tissues or organs of the body, showing nausea, vomiting, headache, etc. [1]. Brain tumors mainly refer to tumors of the nervous system occurring in the skull cavity, including tumors originating from the neuroepithelium, peripheral nerves, meninges and germ cells, lymphoid and hematopoietic tissue tumors, craniopharyngiomas in the sella turcica region, pituitary tumors and granulosa cell tumors, and metastatic tumors. The causes of brain tumors are complex, including environmental factors, air pollution, dietary effects, and other factors [2]. With the development of modern science, electromagnetic waves produced by mobile phones and computers have a certain impact on the occurrence of brain tumors. Air pollution can also induce lung cancer or brain metastasis of lung cancer. Some patients ingest toxic substances to induce brain tumors. In addition, it has a certain relationship with the family heredity of patients. At present, the medical community has not reached a unified standard on the pathogenesis of brain tumors, only pointing out the relevant factors causing such diseases, such as infection, genetics, and carcinogens. However, there is no study to clarify the specific relationship between them and brain tumors [3]. Because the pathogenesis of brain tumors is not clear, there is no specific method to treat brain tumors in clinics. Craniotomy is mainly used for partial resection of tumors. However, craniotomy is an invasive operation, which may lead to various postoperative complications due to various factors [4]. As one of the common complications after craniotomy, intracranial infection will not only prolong the hospital stay, but also increase the medical burden and even threaten the life and health of patients. Therefore, in the early stage of craniotomy, it is of great significance to screen the risk factors of postoperative intracranial infection and take corresponding measures to reduce the incidence of intracranial infection and improve the prognosis [5].

The article "Analysis of the Factors Related to Intracranial Infection after Brain Tumor Surgery" was retracted in 2023. Reasons: unreliable results or conclusions; lack of ethics approval or compliance; concerns about the data; concerns about the peer review.

In order to explore the related factors of intracranial infection after brain tumor surgery, this paper analyzes the clinical application value of a detailed management plan based on the abovementioned risk factors to prevent intracranial infection in patients with brain tumor surgery. Based on this study through the retrospective analysis in January 2020 to December 2020, for 58 cases of brain tumor open-brain surgery patients, the risk factors of postoperative intracranial infection are analyzed, and based on the abovementioned risk factors for the patients with brain tumor open-brain surgery for detail management in order to reduce the incidence of cerebral brain tumor invasive surgery and to provide a theoretical basis.

This paper is organized as follows: Section 22. discusses the related work, followed by the general information in Section 3. The intervention methods and measurement tools are discussed in Section 4, and the experimental results are presented in Section 5. Finally, in Section 6, some concluding remarks are summarized.

## 2. Related Works

For the treatment of brain tumors, craniotomy is a necessary treatment. Intracranial infection is one of the serious complications of brain tumors. The clinical characteristics of craniotomy are often high fever, headache, nausea, and unconsciousness. However, under the shelter of general brain tissue and blood-brain barrier under the skull, the probability of infection is relatively low [6]. However, because the craniotomy of brain tumors is changed to invasive surgery, when the blood-brain barrier is damaged at the same time, it will lead to low immunity. Therefore, foreign microorganisms and bacteria are more likely to invade and cause intracranial infection [7]. Intracranial infection will not only prolong the hospitalization time of patients but also increase the treatment cost. Patients' negative emotions of excessive tension and anxiety before surgery will also reduce the follow-up treatment compliance, resulting in a poor prognosis [8]. Therefore, it is of great significance to explore the relevant risk factors of intracranial infection in patients with brain tumors after surgery and conduct corresponding detailed management according to the abovementioned risk factors [9].

The article "Analysis of the Factors Related to Intracranial Infection after Brain Tumor Surgery" was retracted in 2023. Reasons: unreliable results or conclusions; lack of ethics approval or compliance; concerns about the data; concerns about the peer review.

As a metabolic disease, long-term hyperglycemia will lead to chronic damage and dysfunction of various tissues and nerves, resulting in a certain impairment of the immune function, thus increasing the risk of intracranial infection [10]. The duration of surgery is another risk factor for intracranial infection. Kaewborisutsakul et al. [11] indicated that the probability of intracranial infection in patients with surgery duration ≥5 h is 3 times higher than that in patients with surgery duration <5 h, which is similar to the results of this study. Due to the long operation time, the exposure time of the surgical wound to the air also increases. Therefore, microorganisms and bacteria in the air are more likely to invade, resulting in an increase in the postoperative infection rate [12]. Analysis showed that excessive intraoperative blood loss led to a sharp decline in the number of white blood cells in the blood. The reduction of the immune system function leads to the inability to resist the invasion of foreign bacteria. The occurrence of postoperative intracranial infection or other infection complications is also closely related to the actual situation of patients, and the nursing ability and experience of nursing staff. It is necessary to manage the risk factors in detail and observe their actual effect in clinical application [13].

Detailed management based on risk factors can significantly reduce the incidence rate of intracranial infection in postoperative patients. The analysis shows that because hyperglycemia is a risk factor of intracranial infection, preoperative drug control of hyperglycemia patients can effectively reduce the hyperglycemia environment of patients. This can effectively improve the immune capacity of the immune system and reduce the incidence of postoperative brain infection [14]. Details management during operation includes the following: ensuring the integrity of the operation can reduce unnecessary personnel flow and the number of operating room doors. The switch in the operating room door will cause the surrounding air to enter the operating room, causing bacteria in the operating environment and increasing the risk of cross infection. Medical staff will carry a small amount of bacteria during walking, which will also affect the air quality of the operating room and increase the risk of infection during the operation. Therefore, strict disinfection of surgical equipment and complete appliances before surgery can minimize the mobility of the staff and avoid unnecessary infection [15]. In addition, attention should be paid to the role of psychological intervention in detail management. In order to improve patients' confidence in the prognosis and treatment, the popularization of preoperative health education can help patients cope with complications with a calm attitude [16]. Wang et al. [17] pointed out that being too old also affects the risk factors of intracranial infection in patients with brain tumors after surgery. For the elderly patients with brain tumors, the functions of all aspects of the body have declined to varying degrees, and whether the body can withstand craniotomy is worth careful evaluation.

The article "Analysis of the Factors Related to Intracranial Infection after Brain Tumor Surgery" was retracted in 2023. Reasons: unreliable results or conclusions; lack of ethics approval or compliance; concerns about the data; concerns about the peer review.

## 3. General Information

A retrospective analysis is performed on 58 patients who underwent craniotomy for brain tumor in our hospital from January 2020 to December 2020. According to whether intracranial infection occurred after operation, they are divided into the infection group (*n* = 21) and noninfection group (*n* = 37). In addition, 64 patients who are diagnosed with brain tumor and underwent craniotomy in our hospital from January 2021 to February 2022 are selected and divided into the management group and control group according to the random number table method. There are 32 patients in each group. The management group included 13 females and 19 males, aged from 41 to 58 years, with an average of 51.23 ± 7.34 years, and the course of the disease is 2–5 years. The mean is 4.02 ± 0.82 years; the control group included 16 females and 116 males, aged from 40 to 58 years, with an average of 51.46 ± 7.16 years, and the course of the disease is 2–5 years, with an average of 4.06 ± 0.87)years. There is no statistical difference in general data between the two groups (*P* > 0.05), indicating comparability. All the enrolled patients signed informed consent, and the nursing intervention plan adopted in this study is clinically safe. In the process of this study, the original data (including the test sheet) belong to the research group, but we will protect patients' privacy, no matter what, the patients' name will not appear in the public publications; if the relevant departments need them, they have the right to use these data; the participation of patients is entirely voluntary. The patients have the right not to participate in this study or to withdraw at any time without affecting the normal treatment of the disease. However, we hope to complete this study as far as possible without any special reasons. In any case, the physician must be informed.

The article "Analysis of the Factors Related to Intracranial Infection after Brain Tumor Surgery" was retracted in 2023. Reasons: unreliable results or conclusions; lack of ethics approval or compliance; concerns about the data; concerns about the peer review.

The observation indicators include the following aspects: (1) univariate analysis of risk factors for intracranial infection in postoperative patients with brain tumor; (2) the binary logistic regression model is used to analyze the risk factors of intracranial infection after brain tumor surgery. (3) The cases of intracranial infection after different nursing intervention are compared; (4) SAS and SDS scores are compared before and after intervention; (5) the nursing satisfaction rate is investigated.

## 4. Intervention Methods and Measurement Tools

### 4.1. Self-Rating Anxiety Scale

The Self-Rating Anxiety Scale (SAS) is used to evaluate the degree of psychological anxiety of patients and the changes in the treatment process, which score the patients' anxiety, fear, , breathing, and other conditions. The scoring system adopts a 4-level score, and no or little anxiety is recorded as 1 point. A small amount of time is 2 points; most of the time, 3 points; most or all of the time is 4 points. The total score below 50 is normal, 50–70 is classified as anxious state, and over 70 is classified as severe anxiety state.

### 4.2. Self-Rating Depression Scale (SDS)

This scale is used to reflect patients' depression and the changes in the treatment process, including 20 items such as depression, easy to cry, and sleep disorder. The scoring system adopts a 4-level scoring system, among which 10 items are positive scoring and the other 10 items are reverse scoring. A score below 53 indicates normal, between 53 and 72 indicates depression, and a score above 72 indicates major depression. The scores are positively correlated with the degree of depression.

### 4.3. Intervention Methods

The methods of routine intervention in the control group mainly include the following aspects: (1) preoperative knowledge education for patients, including the popularization of craniotomy for brain tumor and possible postoperative complications; (2) strictly disinfect the operating room environment, adjust the temperature and humidity in the operating room according to the differences in patients' physical conditions, and ensure that the operation process is carried out under aseptic conditions; (3) strictly monitor patients' vital characteristics after surgery, observe whether patients have frequent vomiting, blurred consciousness, and other symptoms, and timely report adverse reactions to doctors and take corresponding measures; (4) dredge the patient's trachea in time and remove secretions in the respiratory tract to prevent respiratory dysfunction and avoid infection.

For the management group, based on the detailed management of the risk factors of intracranial infection after brain tumor surgery, the solutions proposed mainly include the following aspects: (1) the clinical data of patients with preoperative analysis and personal information, if patients has high blood sugar, high blood pressure, and other chronic diseases, adopt corresponding measures and drug control their blood sugar and blood pressure in the normal range; (2) implement psychological intervention in patients with the management group, with most patients, the postoperative adverse complications can affect the health and life quality of life, therefore, the preoperative complications include depression, anxiety, and other emotions. Based on this, the medical staff should handle patients according to preoperative and postoperative complications that may occur and teach them coping styles and explain the cases of successful operation in order to reduce the patient's bad mood, thus improving the confidence of patients for postoperative rehabilitation; (3) the patient's vital signs for changes must be closely monitored strictly in accordance with relevant provisions of the operation process with the doctor, active bleeding in operation must be taken, by observing the patient's facial expression change, assess whether it has the physical discomfort, and shorten the operation time as much as possible to reduce the time the wound is exposed to the air, so as to reduce the infection rate; (4) ensure a complete range of intraoperative surgical supplies, reduce the need to open the surgical door multiple times due to the lack of surgical instruments; (5) compress the puncture site for about 30 minutes after surgery, and instruct the patient to keep the head stable as far as possible, do not shake frequently. Monitor the bleeding situation of the wound of the patient closely and treat the bleeding as soon as possible or use hemostatic drugs.

The article "Analysis of the Factors Related to Intracranial Infection after Brain Tumor Surgery" was retracted in 2023. Reasons: unreliable results or conclusions; lack of ethics approval or compliance; concerns about the data; concerns about the peer review.

### 4.4. Criteria for Intracranial Infection

Criteria for intracranial infection depends on the following symptoms: (1) postoperative high fever, temperature test >38.5°C, and headache symptoms; (2) white blood cell count in cerebrospinal fluid >10 × 10^6^/L and peripheral blood white blood cell technique >10 × 10^9^/L; (3) protein quantification > 0.45 g/L and CSF glucose quantification <2.5 mmol/L; (4) bacterial culture specimens of cerebrospinal fluid are positive. If any of the following items 1–3 or 4 is satisfied, it can be determined as intracranial infection.

### 4.5. Satisfaction Survey

This scale compares the nursing satisfaction of the two groups of patients by oral inquiry of nursing staff, and the satisfaction is divided into dissatisfied, general, satisfied, and very satisfied. The satisfaction rate can be calculated by the following formula: satisfaction rate = (very satisfied + satisfied)/number of patients × 100%.

### 4.6. Statistical Processing

SPSS 25.0 statistical software is used for data analysis, and the specific steps include the following: (1) measurement data: the normality test is performed on the data first. If the data followed normal distribution and homogeneity of variance, it is represented by mean ± standard deviation. The paired sample *t* test is used for test within the group. (2) Count data: descriptive statistical analysis is conducted by percentage, and *x*2 test is performed. (3) Multivariate analysis: logistic regression is used to analyze the risk factors of intracranial infection after brain tumor surgery. The abovementioned data show a significant difference with *P* < 0.05. The flow chart of the detailed management scheme is shown in Figure 1.

## 5. Experimental Results

### 5.1. Univariate Analysis of Risk Factors for Intracranial Infection after Cranial Surgery

Table 1 shows the univariate analysis. It can be clearly seen that diabetes mellitus, intraoperative blood loss, and operation time are the related factors for postoperative intracranial infection in patients with brain tumor (*P* < 0.05).

### 5.2. Multivariate Analysis of Risk Factors for Intracranial Infection after Cranial Surgery

The multifactor assignment is shown in Table 2. The occurrence of intracranial infection after brain tumor surgery is taken as the dependent variable, and the complications of diabetes, operation time, and intraoperative blood loss are taken as independent variables.  Table 3 shows the multivariate regression analysis. It is clearly evident that the complications of diabetes, operation time >7 h, and intraoperative blood loss ≥220 ml are independent risk factors for the occurrence of intracranial infection after brain tumor surgery (*P* < 0.05).

### 5.3. Comparison of the Cases of Postoperative Intracranial Infection

Table 4 shows the comparison of intracranial infection rates. It is clearly showed the incidence of intracranial infection in the management group is significantly lower than that in the control group (*P* < 0.05).

### 5.4. Comparison of Psychological State Changes before and after Intervention

Table 5 shows the comparison of mood changes. In Table 5, “^*∗*^” indicates that the mood changes after nursing are statistically significant compared with before nursing.  Figure 2 and Figure 3 show the changes of SAS and SDS, respectively. It can be observed that SAS and SDS scores of patients in the two groups show no significant difference before intervention, and the adverse mood is improved after intervention in different ways. Besides, the improvement degree in the management group is significantly better than that in the control group (*P* < 0.05).

The article "Analysis of the Factors Related to Intracranial Infection after Brain Tumor Surgery" was retracted in 2023. Reasons: unreliable results or conclusions; lack of ethics approval or compliance; concerns about the data; concerns about the peer review.

### 5.5. Comparison of Nursing Satisfaction

Table 6 shows the comparison of satisfaction. It is found that nursing satisfaction in the management group is significantly higher than that in the conventional group (*P* < 0.05).

## 6. Conclusion

In order to explore the related factors of intracranial infection after brain tumor surgery, this paper analyzes the clinical application value of the detailed management plan based on the abovementioned risk factors to prevent intracranial infection in patients with brain tumor surgery. Multiple regression showed that complications with basic diabetes, prolonged operation time, and increased blood loss were independent risk factors for postoperative intracranial infection (*P* < 0.05). Experimental results show that in the detail management to control the blood of patients with preoperative complications, at the same time, taking some measures to shorten the operation time to accelerate the process of operation can significantly reduce the occurrence of postoperative intracranial infection in patients. Moreover, psychological intervention can improve the patient's compliance with treatment and treatment confidence, and accelerate the recovery of the disease. In the future, we will systematically analyze and summarize how to care for patients with postoperative intracranial infection and conduct more clinical trials to reduce the risk of intracranial infection.

## Figures and Tables

**Figure 1:** Detail management intervention flow chart.

**Figure 2:** Changes of SAS.

**Figure 3:** Changes of SDS.

**Table 1:** Univariate analysis.

Item	Infection group (*n* = 21)	Uninfected group (*n* = 37)	t/*x*2	*P*
Gender			0.222	0.637
Man	11 (52.38%)	17 (45.95%)		
Woman	10 (47.62%)	20 (54.05%)		
Age (years)	45.12 ± 4.52	46.03 ± 4.62		
Course of the disease (years)	3.48 ± 0.52	3.52 ± 0.48	−0.296	0.768
Diabetes mellitus			6.348	0.012
*Y*	14 (66.67%)	12 (32.43%)		
*N*	7 (33.33%)	25 (67.57%)		
Hypertension			0.803	0.370
*Y*	16 (76.19%)	24 (64.86%)		
*N*	5 (23.81%)	13 (35.14%)		
Amount of bleeding (m)	276.24 ± 29.45	187.34 ± 18.52	14.131	<0.001
Time of operation (hours)	7.52 ± 0.32	6.17 ± 0.47	11.693	<0.001
Tumor location			0.946	0.331
Anterior skull base	13 (61.90%)	18 (48.65%)		
Posterior cranial	8 (38.10%)	19 (51.35%)		
Smoking			0.181	0.671
*Y*	12 (57.14%)	19 (51.35%)		
*N*	9 (42.86%)	18 (48.65%)		

**Table 2:** Multiple factor assignment.

Variable	Assignment
Dependent variable	
Intracranial infection	*Y* = 1; *N* = 0
Independent variables	
Amount of bleeding (ml)	＞7 = 1; ≤7 = 0
Time of operation (hours)	≥220 = 1;＜220 = 0
Diabetes mellitus	*Y* = 1; *N* = 0

The article "Analysis of the Factors Related to Intracranial Infection after Brain Tumor Surgery" was retracted in 2023. Reasons: unreliable results or conclusions; lack of ethics approval or compliance; concerns about the data; concerns about the peer review.

**Table 3:** Multivariate regression analysis.

Item	B	S.E.	Wald	*P*	Exp (B)	95% CI
Amount of bleeding (ml)	2.132	1.016	4.403	0.003	8.435	1.151∼11.357
Time of operation (hours)	2.398	1.211	3.923	0.019	10.998	6.313∼17.242
Diabetes mellitus	2.952	1.240	5.664	0.004	1.150	0.192∼1.983

**Table 4:** Comparison of intracranial infection rates.

Group	Number	Number of cases of intracranial infection	Intracranial infection rate
Management group	32	3	9.38%
Control group	32	10	31.25%
*x* ^*2*^			4.730
*P*			0.030

**Table 5:** Comparison of mood changes.

Group	Number	SAS		SDS	
		Before the intervention	After the intervention	Before the intervention	After the intervention
Management group	32	76.63 ± 1.24	26.65 ± 1.09^*∗*^	71.19 ± 1.03	27.79 ± 1.26^*∗*^
Control group	32	75.58 ± 1.21	33.37 ± 1.17^*∗*^	72.21 ± 1.06	38.86 ± 1.21^*∗*^
*T*		0.163	−2.547	−0.077	−3.465
*P*		0.871	0.013	0.939	0.001

**Table 6:** Comparison of satisfaction.

Group	Number	Dissatisfied	General	Satisfied	Very satisfied	Satisfaction
Management group	32	0 (0.00%)	2 (6.25%)	9 (28.13%)	21 (65.63%)	30 (93.75%)
Control group	32	1 (3.13%)	7 (21.88%)	10 (31.25%)	14 (43.75%)	24 (75.00%)
x2						4.267
*P*						0.039

## Data Availability

The simulation experiment data used to support the findings of this study are available from the corresponding author upon request.
